The article "Mechanism of Action of Yin Nourishing and Heat Clearing Prescription in Treating Cough Variant Asthma Based on Network Pharmacology and Molecular Docking Verification" was retracted in 2023. Reasons: unreliable results or conclusions; concerns about the data; concerns about the peer review; concerns about the citations.

# Mechanism of Action of Yin Nourishing and Heat Clearing Prescription in Treating Cough Variant Asthma Based on Network Pharmacology and Molecular Docking Verification

**DOI:** 10.1155/2022/7518109

**Published:** 2022-07-12

**Authors:** Yin Zhang, Yixin Cui, Qi Chen, Fagen Li, Shaodan Li

**Affiliations:** Department of Traditional Chinese Medicine, The Sixth Medical Center, General Hospital of Chinese PLA, Beijing 100853, China

## Abstract

**Objective:**

To explore the mechanism of action of the yin nourishing and heat clearing prescription in treating cough variant asthma (CVA) based on network pharmacology (NP).

**Methods:**

The active ingredients and targets of the yin nourishing and heat clearing prescription were screened using the Traditional Chinese Medicine System Pharmacology Analysis Platform (TCMSP); CVA targets were screened by the GeneCards, NCBI gene, and OMIM databases to construct the component-target network and the protein-protein interaction (PPI) network. GO functional enrichment analysis and Kyoto Encyclopedia of Genes and Genomes (KEGG) pathway enrichment analysis of the target genes were performed to construct the component-disease-pathway-target biological network. Moreover, CVA-related core target structures with high values were subjected to molecular docking (MD) with the active components.

**Results:**

We found 265 eligible targets in the prescription and 1115 CVA-related genes. The medicine targets were intersected with disease targets, which yielded 148 common targets. After topology analysis, 66 key targets were screened. Upon GO functional annotation, 2408 biological processes, 153 molecular functions, and 162 KEGG pathways were enriched. Molecular docking results suggested that the major active ingredients of the prescription showed high affinity to the key targets, among which AKT1 might be the most important target.

**Conclusions:**

Active ingredients might act on AKT1, IL-6, VEGFA, IL-1B, and JUN to suppress eosinophil accumulation, decrease histamine release, suppress airway inflammation, regulate the airway immune microenvironment, increase autophagy in lung tissue, inhibit mucus production, and reduce airway resistance and hyperresponsiveness, thus treating CVA. Our findings provide a reference for further research and clinical applications of the prescription.

## 1. Introduction

Cough variant asthma (CVA) is a special type of asthma with repeated chronic persistent dry cough as the sole or major clinical manifestation. The symptom usually lasts for 8 weeks or longer, and it is closely related to classic asthma (CV). Generally, CVA is the precursor of CV, and about 35.7% of CVA cases will develop into CV within 5 years [1], severely affecting human health. CVA is characterized by airway hyperresponsiveness (AHR), airway eosinophil inflammatory infiltration, tissue remodeling, and excessive mucus secretion, accompanied by cough sensitivity [2]. The existing western CVA treatment guidelines recommend inhalation of bronchodilators and corticosteroids as the initial therapeutic regimen [3]. However, large-dose inhaled bronchodilators and corticosteroids may result in multiple side effects such as vascular remodeling [4]. Moreover, the long-term use of these agents may induce lung dysfunction or other adverse reactions, and the disease is likely to recur after drug withdrawal. By contrast, traditional Chinese medicine (TCM) exhibits distinct advantages and characteristics in treating CVA [5]. We applied a yin nourishing and heat clearing prescription in treating CVA and obtained favorable clinical efficacy. Based on network pharmacology (NP) analysis and molecular docking (MD) simulations, we constructed a drug-active ingredient-target-disease interaction network, and we illustrate the possible mechanism of action of the yin nourishing and heat clearing prescription in treating CVA, so as to provide a theoretical foundation for future basic studies.

The article "Mechanism of Action of Yin Nourishing and Heat Clearing Prescription in Treating Cough Variant Asthma Based on Network Pharmacology and Molecular Docking Verification" was retracted in 2023. Reasons: unreliable results or conclusions; concerns about the data; concerns about the peer review; concerns about the citations.

## 2. Materials and Methods

### 2.1. Research Objects

The active ingredients (compounds) and targets of medicines contained in the yin nourishing and heat clearing prescription (Beishashen, Maidong, Zhimu, Huangqin, Qianhu, and Xingren), the targets of CVA, and the molecular mechanism underlying the effects of the yin nourishing and heat clearing prescription in treating CVA were studied.

### 2.2. NP Research of the Yin Nourishing and Heat Clearing Prescription

The components of the yin nourishing and heat clearing prescription were searched against the TCMSP database to predict the targets. In addition, the GeneCards, NCBI gene, and OMIM databases were searched to screen CVA targets. A Venn diagram was generated to obtain the targets of the yin nourishing and heat clearing prescription in treating CVA. Thereafter, the protein-protein interaction (PPI) network of common targets between the prescription and CVA was constructed based on the String database, and the constructed PPI network was analyzed with related parameters. Afterward, topology analysis was conducted with the NetworkAnalyzer tool to screen the core targets of the yin nourishing and heat clearing prescription in treating CVA. A compound-disease-target regulatory network was constructed using Cytoscape 3.8.0. The core targets were selected to conduct Gene Ontology (GO) functional annotation and Kyoto Encyclopedia of Genes and Genomes (KEGG) pathway enrichment analyses to construct the component-disease-pathway-target network (Figure 1).

The article "Mechanism of Action of Yin Nourishing and Heat Clearing Prescription in Treating Cough Variant Asthma Based on Network Pharmacology and Molecular Docking Verification" was retracted in 2023. Reasons: unreliable results or conclusions; concerns about the data; concerns about the peer review; concerns about the citations.

### 2.3. Screening of Effective Components and Targets of the Yin Nourishing and Heat Clearing Prescription

Eligible candidate compounds and corresponding targets were screened against the TCMSP database [6] (https://tcmspw.com/tcmsp.php) using the terms “Beishashen,” “Lugen,” “Huangqin,” “Lianqiao,” “Qianhu,” and “Xingren,” with oral bioavailability ≥ 30% and drug likeness ≥ 0.18 as the criteria. Then, the targets were corrected based on the UniProt database (https://www.uniprot.org/) [7], where the species was restricted to “*Homo sapiens*,” and the targets were converted to corresponding genes.

### 2.4. Screening of CVA-Related Targets

Human genes were retrieved from the GeneCards database [8] (https://www.genecards.org/), the NCBI gene database [9] (https://www.ncbi.nlm.nih.gov/), and the OMIM database [10] (https://www.omim.org/), using the keyword “cough variant asthma.” Targets obtained from the GeneCards database were screened by the median score, so as to obtain the more relevant targets.

### 2.5. Prediction of Potential Targets of the Yin Nourishing and Heat Clearing Prescription in Treating CVA

The targets of the effective components of the prescription and CVA-related targets were imported into the Venn diagram plotting software Venny 2.1. The intersection was taken as potential targets of the prescription in treating CVA.

### 2.6. Construction of the PPI Network

The common drug-disease targets were imported into the String database [11] (https://string-db.org/cgi/input.pl), where the research species was restricted to “*Homo sapiens*,” the minimum interaction score was set to the median confidence (0.400), and the remaining parameters were set at default values for the construction of the PPI network.

### 2.7. Topology Analysis

The PPI network was imported into Cytoscape 3.8.0 software [12] for topology analysis with the NetworkAnalyzer tool. Genes with degree values greater than average were selected as the key targets.

### 2.8. Construction of the Component-Disease-Target Network and Selection of Key Active Ingredients

To better understand the complicated interactions among components, CVA, and the corresponding targets, the component-disease-target network diagram was built based on the enrolled components, disease, and targets, which was later imported into Cytoscape 3.8.0 for plotting the network diagram and for topology analysis.

### 2.9. GO Functional Annotation and KEGG Pathway Enrichment Analysis

The common drug-disease targets were analyzed for GO term enrichment in the biological process (BP), molecular function (MF), and cell component (CC) categories. The terms with *P*_corr_ < 0.05 were screened based on the String database. Later, histograms and bubble charts were plotted using the clusterProfiler, enrichplot, and ggplot2R packages of R 4.0.3 software. Next, the common drug-disease targets were subjected to KEGG pathway enrichment analysis. Based on the String database, terms with *P*_corr_ < 0.05 were screened. Next, histograms and bubble charts were plotted using the clusterProfiler package of R 4.0.3 software, and the top 20 pathways were visualized.

The article "Mechanism of Action of Yin Nourishing and Heat Clearing Prescription in Treating Cough Variant Asthma Based on Network Pharmacology and Molecular Docking Verification" was retracted in 2023. Reasons: unreliable results or conclusions; concerns about the data; concerns about the peer review; concerns about the citations.

### 2.10. Construction of the Component-Disease-Pathway-Target Network

The component-disease-pathway-target network file was imported into Cytoscape 3.8.0 to plot the pathway network diagram, so as to more intuitively exhibit the “multicomponent and multitarget” characteristics of the TCM active ingredients in treating CVA.

### 2.11. MD Simulations

Five key targets were screened, and then, the compound names, molecular weights, and 2D structures of five active ingredients were determined based on the PubChem database (http://pubchem.ncbi.nlm.nih.gov/). Later, the corresponding 3D structures of active ingredients were downloaded from the RCSB PDB database (http://www.rcsb.org/). Next, the ligands and proteins needed for MD were prepared using AutoDock Vina software (http://vina.scripps.edu/). For target proteins, their crystal structures were preprocessed to satisfy the low-energy conformation of the ligand structure. Finally, these five key target structures were molecularly docked with the five active ingredient structures. The affinity (kcal/mol) value represents the binding capacity between the two, with a lower value indicating more stable binding. The top five docking results with the lowest binding energy were selected for plotting. At last, Pymol software was utilized to analyze the docking results.

## 3. Results

### 3.1. Active Ingredients and Targets of the Yin Nourishing and Heat Clearing Prescription

After searching against the TCMSP database, correcting based on the UniProt database, and removing the nonhuman targets and duplicates, there were altogether 24 components and 211 targets for Lianqiao, 1 component and 30 targets for Lugen, 24 components and 179 targets for Qianhu, 8 components and 169 targets for Beishashen, 36 components and 120 targets for Huangqin, 19 components and 68 targets for Xingren, and 16 components and 112 targets for Rhizoma Anemarrhenae. After removing the duplicate targets, we obtained 265 targets in total.

### 3.2. Extraction of CVA Target Genes

In total, 1075 related targets were obtained from the GeneCards database, 16 from the NCBI database, and 60 from the OMIM database. After removing the duplicates, a total of 1115 CVA-related genes were acquired.

The article "Mechanism of Action of Yin Nourishing and Heat Clearing Prescription in Treating Cough Variant Asthma Based on Network Pharmacology and Molecular Docking Verification" was retracted in 2023. Reasons: unreliable results or conclusions; concerns about the data; concerns about the peer review; concerns about the citations.

### 3.3. Potential Targets of the Yin Nourishing and Heat Clearing Prescription in Treating CVA

The screened drug targets were intersected with the disease targets, and after mapping, 148 common targets between the yin nourishing and heat clearing prescription and CVA were obtained, which were imported into Venny 2.1 to plot the Venn diagram (Figure 2). The left circle exhibits the 1115 CVA-related targets and genes, whereas the right panel shows the 265 core targets of the yin nourishing and heat clearing prescription after screening. The intersecting part represents the 148 common targets. These targets were considered candidate drug targets in CVA treatment and subsequently subjected to pathway enrichment analysis.

### 3.4. Construction of the Drug-Active Ingredient-Target Network of the Yin Nourishing and Heat Clearing Prescription

Based on the abovementioned results, the “drug-active ingredient-target” network was constructed with Cytoscape, and the PPI network diagram was plotted (Figure 3). Each node indicates a protein, and each edge represents the relation between an active ingredient and a target. The node color and size were adjusted according to the degree value, with a larger node and darker red color indicating a greater degree value. Each edge represents the relation between a single drug and an active ingredient, as well as the relation between an active ingredient and a target. The thickness of a line indicates the edge betweenness, with a thicker line representing higher betweenness and hence a stronger relation. In the network diagram, 148 targets show protein interactions and 2904 edges represent protein interactions, with an average degree value of 39.2.

### 3.5. Prediction of Core Targets of the Yin Nourishing and Heat Clearing Prescription in Treating CVA

After topology analysis and sorting according to the degree value, altogether 66 genes with degree scores greater than the average were selected as the key targets. The top 20 targets were utilized for plotting using R 4.0.3, with the abscissa indicating the degree value of each target, where a greater number of nodes indicate that the target has a pivotal role in the network and shows a higher probability as a core target. As shown in Figure 4, AKT1, IL-6, VEGFA, IL-1B, and JUN might be the core targets.

### 3.6. Component-Disease-Target Network Diagram

In the plotted component-disease-target network diagram, light purple indicates active ingredients, green represents drug targets acting on the disease, and yellow indicates TCM components (Figure 5).

### 3.7. Screening of Key Components in the Yin Nourishing and Heat Clearing Prescription

The screened active chemical component names were combined with the component MOL IDs (Table 1). They were sorted according to degree value, with a higher degree value indicating higher importance of the component. The top 5 chemical compounds with the highest degree values (Table 1) were used for subsequent analysis. The compound with the highest degree value was quercetin, followed by luteolin, kaempferol, wogonin, and tanshinone IIa. These compounds might be the key compounds of the yin nourishing and heat clearing prescription in treating CVA.

The article "Mechanism of Action of Yin Nourishing and Heat Clearing Prescription in Treating Cough Variant Asthma Based on Network Pharmacology and Molecular Docking Verification" was retracted in 2023. Reasons: unreliable results or conclusions; concerns about the data; concerns about the peer review; concerns about the citations.

### 3.8. GO Enrichment Analysis

The targets were subject to GO functional analysis based on the DAVID database. It was found that among the 148 common targets between the yin nourishing and heat clearing prescription and CVA, 2408 BPs (*P* < 0.01), 153 MFs, and 82 CCs were enriched. These GO terms were sorted according to the *P* value. The top 10 terms from each category were screened as key functional annotations, and the bubble chart was plotted, as shown in Figure 6, where the abscissa indicates the number of enriched genes (also indicated by dot size) and the colored dot indicates the *P* value (the redder the color, the lower the *P* value). The main enriched BPs included response to molecule of bacterial origin, response to metal ion, cellular response to chemical stress, response to oxidative stress, response to drug, cellular response to oxidative stress, reactive oxygen species (ROS) metabolic process, response to ROS, and epithelial cell proliferation. The main enriched CCs were membrane raft, membrane microdomain, membrane region, caveola, plasma membrane raft, vesicle lumen, cytoplasmic vesicle lumen, secretory granule lumen, and apical part of cells. The main enriched MFs were cytokine receptor binding, signaling receptor activator activity, nuclear receptor activity, ligand-activated, transcription factor activity, receptor ligand activity, and DNA-binding transcription factor binding.

### 3.9. KEGG Pathway Enrichment Analysis Results

The drug-disease common targets were subjected to KEGG pathway enrichment analysis. It was found that 148 intersected target genes were significantly enriched in 162 signaling pathways (*P* < 0.05). The top 20 pathways were selected, as shown in Figure 7, where a larger dot indicates that more genes were enriched and red color indicates a lower *P* value. Pathways not related to CVA such as the AGE-RAGE signaling pathway in diabetic complications were excluded. Finally, three pathways were identified, including the PI3K-AKT signaling pathway, the IL-17 signaling pathway, and the TNF signaling pathway. This suggests that the effects of the yin nourishing and heat clearing prescription on CVA are mediated by the above pathways, among which the PI3K-AKT signaling pathway has the most significant effect.

The article "Mechanism of Action of Yin Nourishing and Heat Clearing Prescription in Treating Cough Variant Asthma Based on Network Pharmacology and Molecular Docking Verification" was retracted in 2023. Reasons: unreliable results or conclusions; concerns about the data; concerns about the peer review; concerns about the citations.

### 3.10. Construction of the Component-Disease-Pathway-Target Network

Using the Merge function of Cytoscape 3.8.0, the disease-drug-component-target network was generated, and the pathway network diagram was plotted (Figure 8). In the diagram, compounds are indicated in blue, the targets of TCM in treating CVA are indicated in pink, the 20 most significant pathways are indicated in green, and the main components of the yin nourishing and heat clearing prescription are indicated in purple. TCM components are represented by 7 nodes, the effective components (excluding those not directly connected with targets) are represented by 91 nodes, CVA-related disease targets (excluding free protein points) are represented by 148 nodes, and the CVA target-related pathways are represented by 20 nodes. As observed from the network diagram analysis results, among the effective components, quercetin had the most edges, followed by luteolin, kaempferol, wogonin, and tanshinone IIa. Among the potential targets, AKT1, IL-6, VEGFA, and MAPK3 had the most edges. Of those pathways, the PI3K-AKT, IL-17, and TNF signaling pathways had the most connections with potential targets. Based on the PPI network, the data were analyzed, which uncovered that the AKT1, IL-6, VEGFA, IL-1B, and JUN nodes had significantly higher degree values compared with other targets; therefore, they were predicted as the potential core targets. Figure 8 intuitively presents the “multicomponent and multitarget” characteristics of TCM active ingredients in treating CVA.

### 3.11. MD Results

The top five compounds with the highest degree values screened in Section 2.7 were subjected to MD analysis with the CVA core proteins. Note that a lower affinity value indicates tighter binding. As observed from Figure 9, AKT1 had high docking efficiency with MOL000098, MOL000006, MOL000422, and MOL007154, with values of −9.6 kcal/mol, −9.8 kcal/mol, −9.6 kcal/mol, and−10.4 kcal/mol, respectively. In addition, JUN also had relatively high docking efficiency with MOL007154, with a value of −9.7 kcal/mol. The binding patterns between AKT1 as well as JUN and active ingredients of the yin nourishing and heat clearing prescription are presented in Figure 10.

## 4. Discussion

### 4.1. Theoretical Evidence with respect to the Mechanisms Underlying the Effects of the Yin Nourishing and Heat Clearing Prescription in Treating CVA

CVA is an atypical form of asthma, which is usually caused by stimulating factors such as upper respiratory tract infection, cold air, dust, and unpleasant odor [13]. It is insensitive to antibiotic therapy, and bronchodilators can temporarily relieve the symptoms. CVA shares common features with classical asthma such as eosinophilic inflammation and airway remodeling, but the former does not show typical manifestations of asthma such as wheezing or dyspnea [14], and it is also different from classical asthma in terms of pulmonary function [15]. At present, the pathogenic mechanism of CVA remains unclear. Some research suggests that CVA is related to persistent chronic airway inflammation, airway hyperresponsiveness, neurogenic inflammation, small airway dysfunction, and airway remodeling [16–19]. In clinical settings, bronchodilators, leukotriene receptor antagonists, and glucocorticoids are usually used to treat CVA, but the long-term effect is unsatisfying and the recurrence rate is high. We applied a yin nourishing and heat clearing prescription in clinical practice to treat CVA and obtained a favorable effect [20, 21], based on the understanding of CVA from the perspective of TCM theory as “yin deficiency is the root, and lung heat is the symptom.” CVA is associated with the typical clinical syndrome of yin deficiency cough; the accompanying symptoms including sore throat, pharyngeal itching, foreign body sensation in the throat, tongue coating, and a pulse condition also basically conform to the yin deficiency and internal heat syndrome. Therefore, it is speculated that yin deficiency combined with internal heat is the major pathogenic mechanism of CVA, and yin nourishing and heat clearing can be used as the major treatment for CVA. One study reported that some herbal medicines with yin nourishing and dryness moistening effects can regulate the serum levels of IgE, 25-(OH)-D3, and related inflammatory factors to regulate the immune response, control airway inflammation, and relieve CVA symptoms [22]. Another study suggested that herbal medicines with yin nourishing and dryness moistening effects can downregulate the expression of cytokines like eosinophilic cationic protein (ECP), IL-4, and IL-5 to regulate the inflammatory response and treat CVA [23]. In this study, the yin nourishing and heat clearing prescription mainly consisted of Beishashen, Radix Ophiopogonis, Rhizoma Anemarrhenae, Huangqin, Qianhu, and Xingren. Beishashen is the monarch drug that can nourish yin to clear away lung heat and expel phlegm to arrest coughing. Radix Ophiopogonis can nourish the lungs to clear away heat, and Rhizoma Anemarrhenae can clear away accumulated lung heat with certain nourishing effects, while Huangqin can clear away heat and dry dampness, purge fire, and remove toxins; these three medicines serve as the main drugs, which help to nourish lung yin and clear away lung heat. Meanwhile, Qianhu and Xingren have the effects of depressing qi, resolving phlegm, dispelling wind, and clearing heat. Therefore, all the medicines had the function of lung ventilation and regulation. Based on previous research, it was speculated that this yin nourishing and heat clearing prescription must have therapeutic potential.

The article "Mechanism of Action of Yin Nourishing and Heat Clearing Prescription in Treating Cough Variant Asthma Based on Network Pharmacology and Molecular Docking Verification" was retracted in 2023. Reasons: unreliable results or conclusions; concerns about the data; concerns about the peer review; concerns about the citations.

### 4.2. Possible Mechanism of Action by which Active Ingredients of the Yin Nourishing and Heat Clearing Prescription Treat CVA

In this study, the TCMSP database was utilized to screen the major active ingredients of the yin nourishing and heat clearing prescription with high degree values, including quercetin, luteolin, kaempferol, and tanshinone IIa. Of these, the flavonoid compound quercetin has anti-inflammation and antiallergy effects, which can prevent allergen- and platelet activation factor- (PAF-) induced airway obstruction and hyperresponsiveness [24]. In addition, it downregulates the expression of IL-4, IL-5, and miR-155 to suppress the terminal differentiation and proliferation of eosinophil precursor cells and improve the airway inflammatory environment [25]. Further, it promotes the release of proinflammatory factors such as chemokines, thymic stromal lymphopoietin (TSLP), IL-25, and granulocyte-macrophage colony-stimulating factor (GM-CSF), recruits inflammatory cells within the airway, and regulates the survival periods of different inflammatory cells, thus playing an important role in the asthma-related airway inflammatory response [26]. Kaempferol is a flavonoid with antioxidant and antitumor effects and has been extensively applied in clinical settings [27]. One study revealed that it can weaken the transcription of monocyte chemoattractant protein-1 to inactivate the TNF*α*-induced airway inflammation, thus blocking the eosinophil-airway epithelium interaction, suppressing the accumulation of eosinophils in the airway and lung tissues, and effectively improving allergic and inflammatory airway diseases [28]. Luteolin also belongs to flavonoids. Luteolin has anti-inflammation, antiallergy, and antioxidant activities. Its beneficial effects on airway hyperresponsiveness and lung tissue infiltration have also been verified [29, 30]. Luteolin can suppress the activation of the GABA_A_ receptor (GABA_A_R), inhibit excessive production of mucus by goblet cells in lung tissues, improve airway stenosis, and alleviate airway resistance [31]. Moreover, it activates the PI3K-AKT-mTOR signaling pathway to regulate the Beclin-1-PI3KC3 protein complex in mouse lung tissue, and it inhibits the airway inflammatory response and autophagy in lung tissue [32]. In addition, luteolin also reduces the specific airway resistance in ovalbumin-sensitized guinea pigs and decreases white blood cell recruitment, histamine release, and the activities of phospholipase A2 (PLA2) and eosinophil peroxide (EPO) in bronchoalveolar lavage fluid (BALF) [33]. Tanshinone IIA can exert anti-inflammatory effects through circ-Sirt1 and by inhibiting NF-*κ*B translocation [34]. Further, it also reduces the inflammatory factor levels and suppresses airway hyperresponsiveness to relieve CVA [35]. To sum up, the active components in the yin nourishing and heat clearing prescription might be related to suppressing EPO activity, decreasing the release of airway inflammatory factors, regulating the immune microenvironment, improving the autophagy level in lung tissue, reducing histamine release, and suppressing excessive mucus production to decrease the airway resistance.

The article "Mechanism of Action of Yin Nourishing and Heat Clearing Prescription in Treating Cough Variant Asthma Based on Network Pharmacology and Molecular Docking Verification" was retracted in 2023. Reasons: unreliable results or conclusions; concerns about the data; concerns about the peer review; concerns about the citations.

### 4.3. Key Targets and Pathways of the Yin Nourishing and Heat Clearing Prescription in Treating CVA

Many previous studies have suggested that the PI3K-AKT signaling pathway participates in multiple key steps regulating airway inflammation, excessive mucus secretion, airway epithelial autophagy, and airway remodeling, leading to CVA. For instance, blocking the PI3K-AKT signaling pathway decreases the infiltration of eosinophils, neutrophils, and lymphocytes in lung tissues, thus suppressing airway inflammation and excessive mucus secretion [36, 37]. ROS can activate the PI3K-AKT signaling pathway and transcription factors such as NF-*κ*B and promote the Th2 cell predominant response to aggravate the inflammatory response and stimulate airway smooth muscle cell proliferation as well as excessive mucus secretion [38]. The Lyn kinase can activate the PI3K-AKT signaling pathway to suppress inflammatory cell infiltration in airway tissues of rats, restrain the inflammatory response, and improve excessive mucus secretion [39]. mTOR, a downstream gene of PI3K, is a major suppressing signal of autophagy [40], which can regulate autophagy to modulate the expression of Th1 and Th2 cytokines and the activation of airway epithelial inflammatory cells [41]. AKT kinase is the major intermediate between PI3K kinase and mTOR kinase, which suppresses the phosphorylation of AKT and mTOR and downregulates the PI3K-AKT-mTOR signaling pathway, inhibiting airway epithelial autophagy and thus alleviating airway inflammation [42]. Besides, upregulation of autophagy through the PI3K-AKT signaling pathway and downregulation of the TLR2-PI3K-AKT signaling pathway also alleviated the airway inflammatory response in mice [38]. One study reported that multiple enzymes, including aldose reductase, tyrosine phosphatase 1, and protein kinase C*δ*, can promote airway remodeling via the PI3K-AKT signaling pathway [43]. In this study, KEGG pathway enrichment analysis suggested that 162 pathways, including the PI3K-AKT, IL-17, and TNF signaling pathways, were closely related to CVA occurrence; in particular, the PI3K-AKT signaling pathway had a significant effect. This indeed suggests that the mechanisms underlying the beneficial effects of the components of the yin nourishing and heat clearing prescription in treating CVA may be closely related to the PI3K-AKT signaling pathway. Our MD simulation results confirmed that AKT1, with the most nodes, had the highest affinity for the major active ingredients of the yin nourishing and heat clearing prescription. AKT1 is a widely expressed serine/threonine kinase, and it is also the core protein in the PI3K-AKT signaling pathway. AKT recruitment and phosphorylation can activate multiple downstream effectors like NF-*κ*B and mTOR [44], which can regulate multiple kinase targets via the PI3K-AKT signaling pathway [45]. Therefore, the therapeutic effect of the yin nourishing and heat clearing prescription in treating CVA may be mediated by multiple mechanisms, including inhibition of the PI3K-AKT signaling pathway. The precise mechanisms should be validated in more in-depth studies.

The article "Mechanism of Action of Yin Nourishing and Heat Clearing Prescription in Treating Cough Variant Asthma Based on Network Pharmacology and Molecular Docking Verification" was retracted in 2023. Reasons: unreliable results or conclusions; concerns about the data; concerns about the peer review; concerns about the citations.

## Figures and Tables

**Figure 1:** Schematic diagram of research strategy.

**Figure 2:** Venn diagram showing the relation of targets of the active ingredients of the yin nourishing and heat clearing prescription with CVA-related targets.

**Figure 3:** Drug-active ingredient target intersection network of the yin nourishing and heat clearing prescription.

**Figure 4:** Twenty key proteins determined by network analysis.

**Figure 5:** Drug-component-target-pathway network analysis diagram.

**Figure 6:** Bubble chart showing the GO functional annotations of the yin nourishing and heat clearing prescription in treating CVA.

**Figure 7:** Pathways enriched among the key targets of the yin nourishing and heat clearing prescription in treating CVA.

**Figure 8:** Drug-component-target-pathway network analysis diagram. Notes: blue indicates compounds, pink indicates the targets of TCM in treating disease, green indicates the 20 most significant pathways, and purple indicates TCM components.

**Figure 9:** Heatmap of molecular docking efficiency.

**Figure 10:** Molecular docking of combinations of active ingredients of the prescription and CVA targets with the highest affinity: (a) AKT1 and MOL000098; (b) AKT1 and MOL000006; (c) AKT1 and MOL000422; (d) AKT1 and MOL007154; (e) JUN and MOL007154.

The article "Mechanism of Action of Yin Nourishing and Heat Clearing Prescription in Treating Cough Variant Asthma Based on Network Pharmacology and Molecular Docking Verification" was retracted in 2023. Reasons: unreliable results or conclusions; concerns about the data; concerns about the peer review; concerns about the citations.

**Table 1:** Representative chemical components, component IDs, and corresponding degree values in the yin nourishing and heat clearing prescription.

MOL ID	Name	Degree
MOL000098	Quercetin	94
MOL000006	Luteolin	41
MOL000422	Kaempferol	40
MOL000173	Wogonin	31
MOL007154	Tanshinone IIa	28

## Data Availability

The [DATA TYPE] data used to support the findings of this study are available from the corresponding author upon request.
